The article "Down-regulation of microRNA-320 suppresses cardiomyocyte apoptosis and protects against myocardial ischemia and reperfusion injury by targeting IGF-1" was retracted in 2025. Reasons: plagiarized images; duplicated images; overlap with other authors' work; concerns about the authorship.

# Down-regulation of microRNA-320 suppresses cardiomyocyte apoptosis and protects against myocardial ischemia and reperfusion injury by targeting IGF-1

**DOI:** 10.18632/oncotarget.9240

**Published:** 2016-05-09

**Authors:** Chun-Li Song, Bin Liu, Hong-Ying Diao, Yong-Feng Shi, Ji-Chang Zhang, Yang-Xue Li, Ning Liu, Yun-Peng Yu, Guan Wang, Jin-Peng Wang, Qian Li

**Affiliations:** ^1^ Department of Cardiology, The Second Hospital of Jilin University, Changchun 130041, P. R. China

**Keywords:** microRNA-320, cardiomyocytes, ischemia-reperfusion, hypoxia-reoxygenation, apoptosis rate

## Abstract

Insulin-like growth factor-1 (IGF-1) is an important regulator of cardiomyocyte homeostasis and cardiac structure, and the prosurvival and antiapoptotic effects of IGF-1 have been investigated. However, the effect of microRNA-320 (miR-320) in ischemia and reperfusion (I/R) by targeting IGF-1 is rarely discussed. We investigated the role of miR-320 in I/R injury. A total of 192 healthy female Wistar rats were divided into eight groups (n = 24). Rat heart I/R model was established. Hemodynamics, infarct size weight (ISW), heart function, and rat cardiomyocyte apoptosis were measured. Hypoxia-reoxygenation (H/R) in rat cardiomyocyte was used to simulate the I/R process. The mRNA levels of miR-320 and IGF-1, and proteins levels of IGF-1, IGF-1R, p-IGF-1R, p-ASK1, p-JNK, p-p38, Bcl-2, Bax and Caspase-3 were measured. *In vivo* inhibition of miR-320 expression significantly increased IGF-1 and IGF-1R mRNA levels, elevated the absolute values of SBP, DBP, MAP, ± dp/dtmax, LVEF and LVFS, decreased ISW, LVESD and LVEDd and the number of TUNEL positive cells, lowered the levels of p-ASK1, p-JNK, p-p38, Bax and Caspase-3 and increased expression of Bcl-2 compared to the I/R + NC group. Compared to H/R + NC group *in vitro*, miR-320 inhibition increased IGF-1 mRNA levels, inhibited cardiomyocyte apoptosis, down-regulated p-ASK, p-JNK, p-p38, Bax and Caspase-3 levels, and up-regulated Bcl-2 level. MiR-320 inhibition target elevated IGF-1 mRNA and protein levels, suppress early cardiomyocyte apoptosis of I/R, and inhibited ASK1-JNK/p38 pathway, which provides a new target for clinical study of I/R injury.

## INTRODUCTION

Ischemia/reperfusion (I/R) occur in trauma, vascular reflow, thrombolysis treatment, percutaneous transluminal coronary angioplasty and organ transplantation [1]. Early restoration of blood flow through the occluded coronary artery limitsinfarct size and preserves cardiac function, thereby decreasing mortality [2, 3]. Ischemia induces accumulation of intracellular sodium, hydrogen and calcium ions, resulting in tissue acidosis. Paradoxically, rapid alterations in ion flux and renormalization of pH following reperfusion causes severe cytotoxicity and I/R injury characterized by cell death and functional deterioration as a result of restoration of blood flow [4, 5]. Such I/R injury causes local myocardial inflammation and apoptosis, resulting in irreversible damage to the myocardium [6].

The article "Down-regulation of microRNA-320 suppresses cardiomyocyte apoptosis and protects against myocardial ischemia and reperfusion injury by targeting IGF-1" was retracted in 2025. Reasons: plagiarized images; duplicated images; overlap with other authors' work; concerns about the authorship.

MicroRNAs (miRNAs) play an important role in ischemia preconditioning-mediated cardiac protection by regulating key cellular signaling pathways, making miRNAs the prime therapeutic targets to address myocardial ischemia [7, 8]. For example, miR-92a inhibition using regional locked nucleic acid-92a (LNA-92a) reduces infarct size and post-ischemic loss of function [9]. Similarly, miR-494 activates Akt signaling and targets both pro-apoptotic and anti-apoptotic proteins, leading to cardio-protection against I/R-induced injury [10]. MiR-320 inhibition reduces myocardial I/R injury in mice, and its overexpression increases cardiomyocyte apoptosis and death. However, the cellular pathways stimulated by miR-320 in myocardial I/R injury are currently unknown [11]. Insulin-like growth factor-1 (IGF-1), acts as an essential regulator of cardiac structure, plays an important part in cardiomyocyte homeostasis, such as inhibition of apoptosis, inter alia promotion of cell growth, as well as augmentation of calcium signaling [12]. Indeed, a previous study revealed that IGF-1 facilitated regeneration of infarcted myocardium and also promoted survival of cardiac stem cells [13].

In this study, we investigated the involvement of miR-320 in pathways related to myocardial I/R injury. We also tested for the effects of miR-320 expression on several hemodynamic indexes, myocardial infarct (MI) size and cardiomyocyte apoptosis. A myocardial I/R injury model was successfully induced in rats by occlusion/reperfusion of the left anterior descending coronary artery, and the rats were intramyocardially injected with lentiviral vector encoding miR-320 to study its actions within cardiomyocytes. Finally, we conducted *in vitro* hypoxia-reoxygenation (H/R) experiments using rat cardiomyocytes to simulate I/R and to verify the actions of miR-320 in myocardial I/R injury.

## RESULTS

### MiR-320 binds IGF-1 mRNA and inhibits IGF-1 expression

We found miR-320 binding sites in the 3′UTR of *IGF-1* using thebioinformatics prediction software TargetScan (Figure 1A). In order to verify whether this 3′UTR region of *IGF-1* is indeed targeted by miR-320, wild-type (WT) and mutant reporters were constructed with GV126-IGF-1 3′-UTR. Our results showed that, compared with other groups, co-transfection of miR-320 mimics and recombinant WT GV126-IGF-1 3′-UTR inhibited luciferase activity. Conversely, co-transfection of miR-320 inhibitors and recombinant WT GV126-IGF-1 3′-UTR increased luciferase activity (*P* < 0.05). As expected, co-transfection of miR-320 mimics and recombinant mutant GV126-IGF-1 3′-UTR, co-transfection of miR-320 inhibitors and recombinant mutant GV126-IGF-1 3′-UTR, and co-transfection of miR-320 negative control and recombinant vectors showed no luciferase activity (all *P* > 0.05, Figure 1B). These results suggest that miR-320 binds to *IGF-1* 3′-UTR and inhibits IGF-1 expression.

The article "Down-regulation of microRNA-320 suppresses cardiomyocyte apoptosis and protects against myocardial ischemia and reperfusion injury by targeting IGF-1" was retracted in 2025. Reasons: plagiarized images; duplicated images; overlap with other authors' work; concerns about the authorship.

**Figure 1:** MiR-320 targets *IGF-1* gene **A.** MiR-320 binding sites in the 3′UTR region of *IGF-1* gene detected by TargetScan. **B.** Dual-luciferase reporter gene system showing miR-320 targeting *IGF-1* gene. Different lowercase letters indicate statistically significant differences (*P* < 0.05) with the same letter indicating no difference (*P* > 0.05). Note: miR-320, microRNA-320; *IGF-1*, *Insulin-like growth factor 1*; UTR, untranslated region; wt, wild type; mut, mutant type.

#### Determination of virus transfection efficiency

miR-320 inhibitors lentivirus, miR-320 mimics lentivirus and ad-IGF-1 recombinant adenovirus marked by green fluorescent protein (GFP) that transfected with myocardial tissues of rats were used to observe the expressions of GFP by fluorescence microscopy to determine the transfection efficiency. The virus concentration of effective transfection of myocardial cells was used as the viral effective biological titer, the myocardial cells that were successful transfected showed a green fluorescent virus, and the transfection rates were approximately 85%, 87% and 88%, respectively (Figure 2).

**Figure 2:** Fluorescence detection of 48h in myocardial cells transfected with virus **A.** myocardial cells transfected with miR-320 inhibitors overexpression; **B.** myocardial cells transfected with miR-320 mimics; **C.** myocardial cells transfected with ad-IGF-1.

### MiR-320 and IGF-1 expressions in myocardial tissue and cells

*In vivo* experiments showed that, compared with the sham group, miR-320 expression increased in the I/R, I/R + NC and I/R + ad-IGF-1 groups, suggesting increased miR-320 expression after I/R treatment (all *P* < 0.05). However, there was no difference in miR-320 expression between the I/R, I/R + NC and I/R + ad-IGF-1 groups (all *P* > 0.05). Compared with the I/R, I/R + NC and I/R + ad-IGF-1 groups, miR-320 levels increased remarkably in the I/R + miR-320 mimics + ad-IGF-1 group, but decreased in the I/R + miR-320 inhibitor group (all *P* < 0.05). Compared with sham group, miR-320 levels significantly decreased in sham + miR-320 inhibitor group while increased remarkably in sham + miR-320 mimics + ad-IGF-1 group (both *P* < 0.05) (Figure 3A). Compared with the sham group, IGF-1 mRNA and protein expressions, IGF-1R and p-IGF-1R levels were downregulated in the I/R treated groups (all *P* < 0.05), no significant difference was found among I/R group, I/R + NC group, and I/R + miR-320 mimics + ad-IGF-1 group. And there was no significant difference between I/R + ad-IGF-1 group and I/R + miR-320 inhibitor group (all *P* > 0.05). In comparison with I/R, I/R + NC, and I/R + miR-320 mimics + ad-IGF-1 groups, IGF-1 mRNA and protein expressions and p-IGF-1R levels were markedly increased in the I/R + miR-320 inhibitor group and the I/R + ad-IGF-1 group (all *P* < 0.05). Compared with sham group and sham+ miR-320 mimics+ ad-IGF-1 group, IGF-1 mRNA and protein expressions, IGF-1R and p-IGF-1R levels significantly increased in sham + miR-320 inhibitor group (all *P* < 0.05), while no significant difference was found between sham group and sham + miR-320 mimics + ad-IGF-1 group (*P* > 0.05) (Figure 3B–3D).

The article "Down-regulation of microRNA-320 suppresses cardiomyocyte apoptosis and protects against myocardial ischemia and reperfusion injury by targeting IGF-1" was retracted in 2025. Reasons: plagiarized images; duplicated images; overlap with other authors' work; concerns about the authorship.

**Figure 3:** MiR-320 and *IGF-1* mRNA and protein expressions in myocardial tissue **A–B.** Real time-PCR detecting miR-320 and *IGF-1* mRNA expressions. **C–F.** Western blots detecting IGF-1 protein expression, IGF-1R and p-IGF-1R levels. Different lowercase letters indicate statistically significant differences (*P* < 0.05) with the same letter indicating no difference (*P* > 0.05). Note: miR-320, microRNA-320; *IGF-1*, *Insulin-like growth factor 1*; PCR, polymerase chain reaction.

*In vitro* experiments showed that, compared with the control group, miR-320 expression increased in H/R-treated groups (all *P* < 0.05). MiR-320 mimics increased miR-320 expression in the H/R + miR-320 mimics + ad-IGF-1 group, while miR-320 inhibitors reduced miR-320 expression in the H/R + miR-320 inhibitor group, compared with the H/R, H/R + NC and H/R + ad-IGF-1 groups (all *P* < 0.05). However, there was no significant difference in miR-320 expression among the H/R, H/R + NC and H/R + ad-IGF-1 groups (*P* > 0.05). Compared with control group, miR-320 levels significantly decreased in control + miR-320 inhibitor group while increased remarkably in control + miR-320 mimics + ad-IGF-1 group (both *P* < 0.05) (Figure 4A). In comparison with the control group, IGF-1 mRNA and protein levels were decreased in other H/R treated groups (all *P* < 0.05), while there was no significant difference in IGF-1 expression among the H/R, H/R + NC and HR + miR-320 mimics + ad-IGF-1 groups (all *P* > 0.05). Compared with the H/R, H/R + NC and HR + miR-320 mimics + ad-IGF-1 groups, IGF-1 mRNA and protein levels were increased in the H/R + miR-320 inhibitor group and the HR + ad-IGF-1 group (all *P* < 0.05). Compared with control group and control + miR-320 inhibitor group, IGF-1 mRNA and protein expressions, IGF-1R and p-IGF-1R levels significantly increased in control + miR-320 inhibitor group (all *P* < 0.05), while no significant difference was found between control group and control + miR-320 mimics+ ad-IGF-1 group (*P* > 0.05) (Figure 4B–4D). Both *in vivo* and *in vitro* experiments show that I/R and H/R treatments can lower the expression of miR-320 while elevating the expression of IGF-1 mRNA and protein levels, further suggesting that miR-320 inhibits the expression of IGF-1 mRNA and protein levels.

The article "Down-regulation of microRNA-320 suppresses cardiomyocyte apoptosis and protects against myocardial ischemia and reperfusion injury by targeting IGF-1" was retracted in 2025. Reasons: plagiarized images; duplicated images; overlap with other authors' work; concerns about the authorship.

**Figure 4:** MiR-320 and *IGF-1* mRNA and protein expressions in rat myocardial cells **A–B.** Real time-PCR detecting miR-320 and IGF-1 mRNA expressions. **C–F.** Western blots detecting IGF-1 protein expression, IGF-1R and p-IGF-1R levels. Different lowercase letters indicate statistically significant differences (*P* < 0.05) with the same letter indicating no difference (*P* > 0.05). Note: miR-320, microRNA-320; *IGF-1*, *Insulin-like growth factor 1*; PCR, polymerase chain reaction.

#### Hemodynamic index changes in rat I/R process

We measured several hemodynamic indexes, namely systolic blood pressure (SBP), diastolic blood pressure (DBP), mean arterial pressure (MAP) and ± dp/dt_max_, at various time points (30 min, 1 hr and 2 hrs), finding no significant differences in their values among the analyzed groups before ischemia treatment. With the exception of the sham group, the absolute values of the measured hydrodynamic indexes in I/R treated groups after reperfusion were lower than the baseline values for all time points (all *P* < 0.01), suggesting successful induction of I/R. The absolute values of SBP, DBP, MAP and ± dp/dtmax were higher in the I/R + miR-320 inhibitor and I/R + ad-IGF-1 groups compared with the I/R, I/R + NC and I/R + miR-320 mimics + ad-IGF-1 groups at each time point (all *P* < 0.01). However, no significant difference in hemodynamic indexes was observed among the I/R, I/R + NC and I/R + miR-320 mimics + ad-IGF-1 groups at any time point (all *P* > 0.05). The absolute values of SBP, DBP, MAP and ± dp/dtmax in sham + miR-320 inhibitor group were significantly higher than those in the same time point of sham group and sham + miR-320 mimics + ad-IGF-1 group (*P* < 0.01), while no significant difference was found in each index of different time points between sham group and sham+ miR-320 mimics+ ad-IGF-1 group (*P* > 0.05) (Figure 5). These results indicate that inhibition of miR-320 may target *IGF-1* to improve the hemodynamic index disorder.

**Figure 5:** Hemodynamic changes during ischemia and reperfusion in each group Hemodynamic changes during I/R in the sham, I/R, IR + NC, I/R + miR-320 mimics + ad-IGF-1, I/R + miR-320 inhibitor and I/R + ad-IGF-1 groups. Note: I/R, ischemia/reperfusion; NC, negative control; IGF-1, insulin-like growth factor 1.

The article "Down-regulation of microRNA-320 suppresses cardiomyocyte apoptosis and protects against myocardial ischemia and reperfusion injury by targeting IGF-1" was retracted in 2025. Reasons: plagiarized images; duplicated images; overlap with other authors' work; concerns about the authorship.

#### Changes in cardiac function after I/R treatment

Changes in cardiac function after I/R treatment in each group are shown in Table 1. Compared with the sham group, left ventricular ejection fraction (LVEF) and left ventricular fraction shortening (LVFS) of rat myocardial tissue decreased significantly, while left ventricular endsystolic diameter (LVESD) and left ventricular end diastolic diameter (LVEDd) increased significantly in I/R treated groups (all *P* < 0.05). However, there was no statistically significant difference among the I/R, I/R + NC and I/R + miR-320 mimics + ad-IGF-1 groups (all *P* > 0.05); and compared with the I/R, I/R + NC and I/R + miR-320 mimics+ ad-IGF-1 groups, LVEF and LVFS increased while LVESD and LVEDd decreased in the I/R + miR-320 inhibitor and I/R + ad-IGF-1 groups (all *P* < 0.05). LVEF and LVFS remarkably increased while LVESD and LVEDd decreased significantly in sham + miR-320 inhibitor group when compared with sham group and sham + miR-320 mimics + ad-IGF-1 group (all *P* < 0.05), while there was no statistical significance between sham group and sham + miR-320 mimics + ad-IGF-1 group (*P* > 0.05). These results suggest that inhibition of miR-320 may target *IGF-1* to improve the cardiac function after reperfusion.

**Table 1:** Cardiac function changes 2 weeks after I/R treatment in each group

Group	LVEF	LVFS	LVESD	LVEDd
Sham	58.61 ± 10.33^a^	30.92 ± 7.30^a^	3.83 ± 0.09^a^	2.64 ± 0.36^a^
I/R	24.88 ± 3.53^b^	11.65 ± 1.98^b^	5.90 ± 0.22^b^	4.32 ± 0.71^b^
I/R+NC	25.07 ± 3.21^b^	11.11 ± 2.03^b^	6.01 ± 0.25^b^	4.64 ± 0.69^b^
I/R+miR-320 inhibitor	34.45 ± 2.75^c^	16.63 ± 1.45^c^	5.43 ± 0.11^c^	3.69 ± 0.41^c^
I/R+ad-IGF-1	36.18 ± 2.89^c^	17.47 ± 1.53^c^	5.46 ± 0.14^c^	3.88 ± 0.44^c^
I/R+ miR-320 mimics+ ad-IGF-1	25.76 ± 1.29^b^	10.73 ± 1.01^b^	6.11 ± 0.21^b^	4.76 ± 0.99^b^
Sham+ miR-320 inhibitor	67.24±9.17^d^	34.35±8.24^d^	3.22±0.10^d^	2.01±0.32^d^
Sham + miR-320 mimics+ ad-IGF-1	60.59±10.28^a^	31.14±6.81^a^	3.77±0.08^a^	2.83±0.37^a^

Note: Different lowercase letters indicate statistically significant differences (*P* < 0.05) with the same letter indicating no difference (*P* > 0.05). LVEF, left ventricular ejection fraction; LVFS, left ventricular fraction shortening; LVESD, left ventricular end systolic diameter; LVEDd, left ventricular end diastolic diameter; I/R, ischemia/reperfusion; NC, negative control; miR-320, microRNA-320; IGF-1, insulin like growth factor-1.

The article "Down-regulation of microRNA-320 suppresses cardiomyocyte apoptosis and protects against myocardial ischemia and reperfusion injury by targeting IGF-1" was retracted in 2025. Reasons: plagiarized images; duplicated images; overlap with other authors' work; concerns about the authorship.

### Myocardial infarction (MI) size measurement

The body weight (BW), left ventricle weight (LVW), area at risk weight (AARW) and AARW/LVW showed no differences among the I/R treated groups (all *P* > 0.05). The infarct size weight (ISW) and ISW/AARW showed no differences among the I/R, I/R + NC and I/R + miR-320 mimics + ad-IGF-1 groups (*P* > 0.05), but markedly decreased in the I/R + miR-320 inhibitor group and the I/R + ad-IGF-1 group compared with the I/R, I/R + NC and I/R + miR-320 mimics + ad-IGF-1 groups (all *P* < 0.05) (Table 2). These results imply that miR-320 might target *IGF-1* to lower MI size.

**Table 2:** Myocardial infarct size measured in each group

Group	BW (g)	LVW (g)	AARW (g)	AARW/LVW (%)	ISW (g)	ISW/AARW (%)
Sham	387.4 ± 6.9	0.85 ± 0.03	0	0	0	0
I/R	387.2 ± 8.2	0.84 ± 0.02	0.36 ± 0.03	0.42 ± 0.04	0.150 ± 0.034^a^	42.9 ± 5.8^a^
I/R+NC	385.3 ± 3.9	0.83 ± 0.01	0.36 ± 0.01	0.44 ± 0.02	0.143 ± 0.010^a^	40.6 ± 3.4^a^
I/R+miR-320 inhibitor	386.7 ± 5.7	0.84 ± 0.04	0.36 ± 0.02	0.44 ± 0.03	0.087 ± 0.020^b^	27.7 ± 4.7^b^
I/R+ad-IGF-1	384.0 ± 4.5	0.85 ± 0.01	0.38 ± 0.01	0.45 ± 0.01	0.090 ± 0.018^b^	25.7 ± 3.1^b^
I/R+ miR-320 mimics+ ad-IGF-1	387.5 ± 3.9	0.84 ± 0.01	0.37 ± 0.03	0.43 ± 0.02	0.146 ± 0.021^a^	41.6 ± 4.3^a^
Sham+ miR-320 inhibitor	387.5±6.7	0.84±0.03	0	0	0	0
Sham + miR-320 mimics+ ad-IGF-1	387.4±7.1	0.85±0.02	0	0	0	0

Note: Different lowercase letters indicate statistically significant differences (*P* < 0.05) with the same letter indicating no difference (*P* > 0.05). BW, body weight; LVW, left ventricle weight; AARW, area at risk weight; ISW, infarct size weight; I/R, ischemia/reperfusion; NC, negative control; miR-320, microRNA-320; IGF-1, insulin like growth factor-1.

### Myocardial cell apoptosis

In order to further test whether inhibition of miR-320 can target *IGF-1* to reduce myocardial cell apoptosis, we measured apoptosis rates as well as levels of apoptosis-related factors, Bcl-2, Bax and Caspase-3 in rat myocardial tissues and cells. The effect of miR-320 expression on myocardial cell apoptosis after I/R treatment is shown in Figure 6A–6B. Compared with the sham group (apoptosis rate: 5.36 ± 1.01%), TUNEL positive cells increased significantly in the I/R (apoptosis rate: 44.67 ± 1.54%), I/R + NC (apoptosis rate: 46.67 ± 1.81%) and I/R + miR-320 mimics + ad-IGF-1 (apoptosis rate: 45.71 ± 1.39%) groups (all *P* < 0.05), but no significant differences in apoptosis rate were seen among the I/R, the I/R + NC and I/R + miR-320 mimics + ad-IGF-1 groups (all *P* > 0.05). In comparison with the I/R, I/R + NC and I/R + miR-320 mimics + ad-IGF-1 groups, apoptosis rates significantly decreased in the I/R + miR-320 inhibitor and I/R + ad-IGF-1 groups (25.49 ±1.69 % and 26.62 ± 1.22 %, respectively) (all *P* < 0.05). Apoptosis-related proteins Bcl-2, Bax and Caspase-3 in myocardial tissue were detected by western blot analysis (Figure 6C–6F). Compared with the sham group, the anti-apoptotic factor Bcl-2 decreased sharply, while pro-apoptotic Bax and Caspase-3 increased in the I/R, I/R + NC and I/R + miR-320 mimics + ad-IGF-1 groups (all *P* < 0.05), with no significant differences among the groups (all *P* > 0.05). In comparison with the I/R, I/R + NC and I/R + miR-320 mimics + ad-IGF-1 groups, Bcl-2 expression increased and Bax and Caspase-3 expressions decreased in the I/R + miR-320 inhibitor and I/R + ad-IGF-1 groups (all *P* < 0.05). Bcl-2 expression significantly increased and Bax and Caspase-3 expressions decreased in sham + miR-320 inhibitor group when compared with sham group and sham + miR-320 mimics + ad-IGF-1 group (all *P* < 0.05), while there was no statistical significance between sham group and sham + miR-320 mimics + ad-IGF-1 group (*P* > 0.05).

The article "Down-regulation of microRNA-320 suppresses cardiomyocyte apoptosis and protects against myocardial ischemia and reperfusion injury by targeting IGF-1" was retracted in 2025. Reasons: plagiarized images; duplicated images; overlap with other authors' work; concerns about the authorship.

**Figure 6:** Myocardial cell apoptosis rate and apoptosis-related proteins **A–B.** Cell apoptosis rate detected by TUNEL assay. **C–F.** Bcl-2, Bax and Caspase-3 protein expressions detected by western blotting. Different lowercase letters indicate statistically significant differences (*P* < 0.05) with the same letter indicating no difference (*P* > 0.05). Note: TUNEL, transferase-mediated deoxyuridine triphosphate-biotin nick end labeling; Bcl-2, B-cell lymphoma 2; I/R, ischemia/reperfusion; NC, negative control; IGF-1, Insulin-like growth factor 1.

AnnexinV/PI double staining was used to detect apoptosis in rat myocardial cells (Figure 7A–7B). Compared to the control group (9.11 ± 0.62 %), apoptosis was increased after H/R treatment (all *P* < 0.05). The apoptosis rate in the H/R, H/R + NC and H/R + miR-320 mimics + ad-IGF-1 groups showed no significant differences (47.45 ± 2.54% vs. 50.11 ± 2.87% vs. 50.18 ± 2.29%, all *P* > 0.05). Apoptosis rates were lower in the H/R + miR-320 inhibitor (28.45 ± 2.69%) and HR + ad-IGF-1 (27.18 ± 2.17%) groups (all *P* < 0.05) than in the H/R, H/R + NC and H/R + miR-320 mimics + ad-IGF-1 groups. The levels of apoptosis-related factors Bcl-2, Bax and Caspase-3 in rat myocardial cells are shown in Figure 7C–7F. Bcl-2 levels were lower in H/R treated cells (all *P* < 0.05), compared with the control group. On the other hand, Bax and Caspase-3 expressions were higher in H/R treated cells (all *P* < 0.05) than in the control group. Bcl-2 expression was higher while Bax and Caspase-3 expressions were lower in the H/R + miR-320 inhibitor and H/R + ad-IGF-1 groups (all *P* < 0.05) than in the H/R, H/R + NC and H/R + miR-320 mimics + ad-IGF-1 groups. Bcl-2 expression significantly increased and Bax and Caspase-3 expressions decreased in control + miR-320 inhibitor group when compared with control group and control + miR-320 mimics + ad-IGF-1 group (all *P* < 0.05), while there was no statistical significance between control group and control + miR-320 mimics + ad-IGF-1 group (*P* > 0.05). Both *in vivo* and *in vitro* experiments showed that cell apoptosis rates increase after I/R treatment and that inhibition of miR-320 can target *IGF-1*, therebydecreasing myocardial cell apoptosis as well as the expression of pro-apoptosis factors Bax and Caspase-3, while increasing the expression of anti-apoptosis factor Bcl-2.

The article "Down-regulation of microRNA-320 suppresses cardiomyocyte apoptosis and protects against myocardial ischemia and reperfusion injury by targeting IGF-1" was retracted in 2025. Reasons: plagiarized images; duplicated images; overlap with other authors' work; concerns about the authorship.

**Figure 7:** Rat myocardial cell apoptosis rate and apoptosis-related proteins **A–B.** Cell apoptosis rate detected by Annexin V/Propidium iodide apoptosis assay. **C–F.** Bcl-2, Bax and Caspase-3 protein expressions detected by western blotting. Different lowercase letters indicate statistically significant differences (*P* < 0.05) with the same letter indicating no difference (*P* > 0.05). Note: Bcl-2, B-cell lymphoma 2; H/R, hypoxia/reoxygenation; NC, negative control; IGF-1, Insulin-like growth factor 1.

### ASK1-JNK/p38 signaling pathway expression

To test whether miR-320 targets *IGF-1* to activate the ASK1-JNK/p38 signaling pathway and increase myocardial cell apoptosis, we measured cell apoptosis downstream of the ASK1-JNK/p38 signaling pathway. We also measured the protein levels of p-ASK1, p-JNK and p-p38. Compared with the sham group, p-ASK1, p-JNK and p-p38 levels increased in I/R, I/R + NC and I/R + miR-320 mimics + ad-IGF-1 groups (all *P* < 0.05), but no differences were found among the three groups (all *P* > 0.05). Compared with the I/R, I/R + NC and I/R + miR-320 mimics + ad-IGF-1 groups, p-ASK1, p-JNK and p-p38 levels decreased in the I/R + miR-320 inhibitor and I/R + ad-IGF-1 groups (all *P* < 0.05). p-ASK1, p-JNK and p-p38 levels significantly decreased in sham + miR-320 inhibitor group when compared with sham group and sham + miR-320 mimics + ad-IGF-1 group (all *P* < 0.05), while there was no statistical significance between sham group and sham + miR-320 mimics + ad-IGF-1 group (*P* > 0.05) (Figure 8). Compared with the control group, p-ASK1, p-JNK and p-p38 levels were increased in the H/R, the H/R + NC, and H/R + miR-320 mimics + ad-IGF-1 groups (all *P* < 0.05). However, no significant differences in p-ASK1, p-JNK and p-p38 levels were observed among the H/R, H/R + NC and H/R + miR-320 mimics + ad-IGF-1 groups (all *P* > 0.05). In comparison with the H/R, H/R + NC and H/R + miR-320 mimics + ad-IGF-1 groups, p-ASK1, p-JNK and p-p38 levels were lower in the H/R + miR-320 inhibitor and H/R + ad-IGF-1 groups (all *P* < 0.05) (Figure 9). p-ASK1, p-JNK and p-p38 levels significantly decreased in control + miR-320 inhibitor group when compared with control group and control + miR-320 mimics + ad-IGF-1 group (all *P* < 0.05), while there was no statistical significance between control group and control + miR-320 mimics + ad-IGF-1 group (*P* > 0.05). Our results suggest that inhibition of miR-320 might promote *IGF-1* expression and inhibition of the ASK1-JNK/p38 signaling pathway while reducing myocardial cell apoptosis.

The article "Down-regulation of microRNA-320 suppresses cardiomyocyte apoptosis and protects against myocardial ischemia and reperfusion injury by targeting IGF-1" was retracted in 2025. Reasons: plagiarized images; duplicated images; overlap with other authors' work; concerns about the authorship.

**Figure 8:** Western blot analysis of p-ASK1, p-JNK and p-p38 levels in myocardial tissue Different lowercase letters indicate statistically significant differences (*P* < 0.05) with the same letter indicating no difference (*P* > 0.05). Note: p-ASK1, phosphorylated-apoptosis signal-regulating kinase 1; p-JNK, phosphorylated-c-Jun N-terminal kinase; I/R, ischemia/reperfusion; NC, negative control; IGF-1, Insulin-like growth factor 1.

**Figure 9:** Western blot analysis of p-ASK1, p-JNK and p-p38 levels in rat myocardial cells Different lowercase letters indicate statistically significant differences (*P* < 0.05) with the same letter indicating no difference (*P* > 0.05). Note: p-ASK1, phosphorylated-apoptosis signal-regulating kinase 1; p-JNK, phosphorylated-c-Jun N-terminal kinase; H/R, hypoxia/reoxygenation; NC, negative control; IGF-1, Insulin-like growth factor 1.

## DISCUSSION

Recently, strategies to alter microRNA levels to promote favorable disease outcomes have led to a new field of cardiovascular therapeutics [14]. In a previous study, we demonstrated that miR-320 inhibition using antagomir-320 protects the left ventricle from remodeling after I/R injury [15]. Here we further investigated the role of miR-320 in myocardial I/R injury. Our results show that inhibition of miR-320 using a miR-320 inhibitor protects against myocardial I/R injury specifically by suppressing pro-apoptotic pathways and increasing the activation of anti-apoptotic signals.

Our results show that IGF-1 mRNA and protein levels correlate negatively with miR-320 levels, suggesting that IGF-1 mRNA might be an important miR-320 target *in vivo*. Our results confirm that miR-320 directly binds to the 3′-UTR region of *IGF-1* to negatively regulate IGF-1 expression. This suggests upregulation of miR-320 in myocardial microvascular endothelial cells may impair angiogenesis by dysregulating expression of IGF-1 protein and mRNA [16]. Rather than in cardiomyocytes, inflammasome activation in cardiac fibroblasts is definitively associated with the initial inflammatory response after I/R injury, and inflammasomes and the subsequent activation of inflammasomes, which are formed by I/R, leads to interleukin-1β production, leading to inflammatory responses including inflammatory cell infiltration and cytokine expression in the heart [17].

The article "Down-regulation of microRNA-320 suppresses cardiomyocyte apoptosis and protects against myocardial ischemia and reperfusion injury by targeting IGF-1" was retracted in 2025. Reasons: plagiarized images; duplicated images; overlap with other authors' work; concerns about the authorship.

We found that miR-320 inhibitors increase the absolute values for SBP, DBP, MAP and ± dp/dtmax. On the other hand, these indexes are sharply reduced by I/R treatment, which highlight the positive effects of miR-320 inhibition on the recovery of cardiac function. In addition, our cardiac function study showed that LVEF and LVFS increased while LVESD and LVEDd decreased in the I/R + miR-320 inhibitor group, suggesting inhibition of miR-320 may target IGF-1 to improve cardiac function after reperfusion. Particularly, miR-320 was reported to have the potential to target multiple angiogenesis-related genes, such as *Flk-1, VEGF-c, IGF-1, IGF-1R* and *FGFs* [16]. MiR-320 was also shown to be participated in I/R injury and/or remodeling after MI, which was in consistent with the results in this study [11]. In addition, overexpression of miR-320 resulted in the inhibition of cell proliferation, invasion, migration, and tumorigenesis by targeting IGF-1, which further regulated the signaling pathways downstream, such as phosphoInositide-3 kinase/ serine-threonine kinases (PI3K/AKT) and Mitogen-Activated Protein Kinase/ extracellular-response kinase (MAPK/ERK) [18]. Furthermore, a recent study has suggested that miR- 320 could inhibit tumor development and growth through targeting IGF-1, and miR-320 might act as a new effective target for the treatment of cancer [19]. MiR-320 inhibition also decreased ISW and ISW/AARW confirming that miR-320 inhibitors reduce infarct and thereby protect cardiac function. Similarly, Montgomery et al. found that inhibition of miR-208 was also a potent therapeutic target for modulating cardiac function and remodeling [20].

MiR-320 inhibition decreased the rate of cardiomyocyte apoptosis *in vivo* and *in vitro* by increasing Bcl-2 expression and decreasing Bax and Caspase-3 levels. Bcl-2 family proteins are key regulators of apoptosis and include anti- and pro-apoptotic proteins. Marginal changes in anti- and pro-apoptotic protein ratios result in inhibition or promotion of cell death [21]. Cytochrome c release and caspase activation are prevented by Bcl-2, while Bax promotes cytochrome c release and caspase-3 activation [22]. Activated caspase-3 is one of the main mediators of apoptosis, which exerts its effects by cleaving other caspases and the anti-apoptotic protein Bcl-2 [23].

ASK1-JNK/p38 signaling pathways were activated by I/R and H/R treatment but were suppressed by inhibition of miR-320. ASK1 is a mitogen-activated protein kinase (MAPK) [24, 25] whose activation leads to MKK-4/7, MKK-3/6, JNK and p38 MAPK activation [26]. The stress-activated protein kinases p38 MAPK and JNK are activated in response to a variety of stimuli including ROS, hypoxia, pro-inflammatory cytokines, activated Toll-like receptors, transforming growth factor (TGF)-β, aldosterone and ANG II [27]. The ASK1 pathway modulates apoptosis during viral infections [28, 29]. Interestingly, miR-320 inhibitor decreases activation of p-ASK1, p-JNK and p-p38. MiR-320 inhibition thus down-regulates the ASK1-JNK/p38 signaling pathway, thereby inhibiting apoptosis.

The article "Down-regulation of microRNA-320 suppresses cardiomyocyte apoptosis and protects against myocardial ischemia and reperfusion injury by targeting IGF-1" was retracted in 2025. Reasons: plagiarized images; duplicated images; overlap with other authors' work; concerns about the authorship.

IGF-1 might also activate the post-translational modification of Bcl-2 family proteins. Although the mechanistic link between miR-320 and the ASK1-JNK/p38 signaling pathway requires further examination, we hypothesize that IGF-1 increases ASK1 expression to modulate the ASK1-JNK/p38 signaling pathway. IGF-1 is a critical cardiac survival factor that can increase protein metabolism, promote cell growth, and improve myocardial contraction while protecting the heart against ischemia-induced apoptosis [30]. In addition, IGF-I protein appears to be associated with left ventricular hypertrophy and increased heart function after myocardial infarction [31]. IGF-I was also found to improve yak spermatozoa motility and the rate of oocyte cleavage by reducing the rate of spermatozoa apoptosis through modulation the Bax and Bcl-2 expression [32]. Furthermore, IGF-1 activates cyclic AMP response element binding protein via several signaling pathways, including PI3K and p38-MAPK, which play important roles in the anti-apoptotic action of cardiac myocytes [33].

In sum, miR-320 expression worsens myocardial I/R injury, while its inhibition protects against myocardial apoptosis. MiR-320 inhibition suppresses apoptosis effect mainly via the IGF-1 pathway, affecting the levels of anti-apoptotic Bcl-2 and pro-apoptotic Bax and caspase-3, and inactivating the ASK1-JNK/p38 signaling pathways. This suggests miR-320 may represent a valuable tool and potential therapeutic target for protection against I/R induced cardiac injury.

## MATERIALS AND METHODS

### Dual-luciferase reporter assay

Bioinformatics software such as TargetScan, PicTar and microRNA.org were employed to predict possible targets of rno-miR-320. The *IGF-1* gene was identified as a target and the entire *IGF-1* gene 3′ untranslated regions (UTR) was amplified and cloned into the multiple cloning sites downstream of the GV126 Luciferase gene (Promega Corporation, Madison, WI, US). Based on the predicted target binding site of rno-miR-320 and the *IGF-1* gene, site-directed mutagenesis was employed to abolish the biding site and this mutant was used as a control. A renilla luciferase containing plasmid with thymidine kinase promoter (pRL-TK vector, TaKaRa, Japan) was used as a reporter control to adjust for transfection efficiency. MiR-320 mimics, miR-320 inhibitors and a negative control (NC) were respectively co-transfected with the luciferase reporter vector into HEK293 cells. Luciferase assays were conducted according to dual luciferase assay kit protocol (Promega Corporation, Madison, WI, US). HEK293 cells were purchased from Basic Research Institute of Peking Union Medical College Hospital. The use of cells was added with myllicin to culture in dulbecco's minimum essential medium (DMEM) culture medium with 10% calf serum, and placed it in the incubator with a volume fraction of 5% CO_2_ at 37°C. The liquids were replaced every 2 days and then be digested with 0.25% trypsase and subcultured when the cells grew to 70%~80% of the bottle of culture bottle.

The article "Down-regulation of microRNA-320 suppresses cardiomyocyte apoptosis and protects against myocardial ischemia and reperfusion injury by targeting IGF-1" was retracted in 2025. Reasons: plagiarized images; duplicated images; overlap with other authors' work; concerns about the authorship.

### Experimental animals

A total of 192 female Wistar rats (weight, 320g-350g; age, 12-16 weeks) were purchased from the animal experimental center of the Second Hospital of Jilin University. The temperature of vivarium was set to ~25°C and the humidity was maintained at 60%. Photoperiod was set to 12 hours to mimic the normal physiological day-night cycle. Drinking water and standard forage were available to animals after sterilization. This study was conducted in strict accordance with the recommendations in the Guide for the Care and Use of Laboratory Animals of the National Institutes of Health [34]. This study's protocols were approved by the ethics committee of animal experimental center of the Second Hospital of Jilin University.

### Grouping

The 192 rats were randomly allocated into eight groups (n = 24). 1) Sham group: the heart was exposed after left thoracotomy. The suture line was placed under the left anterior descending artery (LAD) and the coronary artery was not ligated. The whole process lasted 150 min. 2) I/R group: LAD was ligated reversibly and ischemia was induced for 30 min and reperfusion for 120 min. 3) I/R + NC group: seven days after the rats were intramyocardially injected with empty virus expressing GFP, LAD was ligated reversibly. Ischemia was induced for 30 min and reperfusion for 120 min. 4) I/R + miR-320 inhibitors group: seven days after the rats received intramyocardial injection of lentivirus carrying miR-320 inhibitors, I/R was induced as above. 5) I/R + ad-IGF-1 group: ad-IGF-1 recombinant adenovirus was directly injected to the myocardium, and 7 days later LAD was ligated reversibly. Ischemia was induced for 30 min and reperfusion for 120 min. 6) I/R + miR-320 mimics + ad-IGF-1 group: miR-320 mimics and ad-IGF-1 recombinant adenovirus were directly injected to the myocardium, and 7 days later LAD was ligated reversibly. Ischemia was induced for 30 min and reperfusion for 120 min. 7) Sham + miR-320 inhibitors group: suture line was placed under the LAD, the coronary artery was not ligated, and the rats received intramyocardial injection of lentivirus carrying miR-320 inhibitors. 8) Sham + miR-320 mimics+ ad-IGF-1 group: suture line was placed under the LAD, the coronary artery was not ligated, and the rats received intramyocardial injection of lentivirus carrying miR-320 inhibitors and ad-IGF-1. MiR-320 mimics synthesized by chemical methods stimulated endogenous miR-320 expression *in vivo* and enhanced endogenous miR-320 function. MiR-320 inhibitors are chemically modified to inhibit miR-320. Twelve rats in each group were sacrificed at the time of coronary artery flow of 120 min, and then the hearts of rats were taken for the next experiment. In addition, 12 rats in each group were used for the detection of cardiac function after 2 weeks. MiR-320 inhibitor lentivirus marked by GFP, miR-320 mimic lentivirus, empty viral vectors and ad-IGF-1 recombinant adenovirus (titer: 4.0×10^8^pfu/ml) were purchased from Shanghai genechem Gene Technology Co., Ltd.

The article "Down-regulation of microRNA-320 suppresses cardiomyocyte apoptosis and protects against myocardial ischemia and reperfusion injury by targeting IGF-1" was retracted in 2025. Reasons: plagiarized images; duplicated images; overlap with other authors' work; concerns about the authorship.

### Virus vector transfection

Rats were anesthetized with 1.5% pentobarbital sodium (50 mg/kg) and fixed after weighing. Rats were placed immediately on a Harvard rodent ventilator (tidal volume 2–3 mL, respiratory rate 60 per min). Chest skin was sterilized by iodophor after dehairing. Tissue and muscle were bluntly isolated after the skin was cut obliquely. Ribs 3 and 4 were cut longitudinally and the pericardium was cut open to expose the heart. A total volume of 200 μl virus solution was injected using a sterile micro syringe at four different points into the rat left ventricular anterior walls [35, 36]. The chest was closed layer by layer after the surgery. Rats were observed for 30 min for spontaneous breathing and intubation of trachea was removed after stable respiration was achieved and the rats continued feeding for 7 days. An amount of 100,000 U/(per rat per day) penicillin was intraperitoneally injected for 3 days after surgery. MiR-320 mimics sequence: 5′-AAAAGCUGGGUUGAGAGGGCGA-′3, miR-320 inhibitors sequence: 5′-UCGCCCUCU CAACCCAGCUUUU-′3 (Shanghai GenePharma Co., Ltd., Shanghai, China).

### Rat myocardial I/R model establishment

The heart was exposed after a left thoracotomy as described before. A 4-0 suture line loop and a plastic pipe were used to ligate the 2 mm part near the LAD before thoracic cavity was closed to create ischemia. A successful coronary artery ligation was verified by the ST-segment elevation observed in the electrocardiogram and myocardial tissue under the ligation line turned brick-red or pale. After LAD ligation for 30 min, the plastic pipe was removed for reperfusion. The rats in each group used to test for hemodynamic changes and cardiac function were kept alive with their chest closed after I/R treatment, while other rats were sacrificed to obtain specimen for other tests. The body weight (BW) was measured before the rats were sacrificed. Rats were sacrificed 120 min after reperfusion and the heart was collected. In the sham group, the suture line was placed under the LAD and no ligation was made. The sham operation lasted for 150 min and rats were sacrificed to collect the hearts.

The article "Down-regulation of microRNA-320 suppresses cardiomyocyte apoptosis and protects against myocardial ischemia and reperfusion injury by targeting IGF-1" was retracted in 2025. Reasons: plagiarized images; duplicated images; overlap with other authors' work; concerns about the authorship.

### Hemodynamic change

An artery catheter was placed into the left ventricle at the beginning of the I/R process and hemodynamic changes at each time period of the I/R process were recorded using Medlab biological signal acquisition system (Nanjing medease science and technology co., Ltd). Systolic blood pressure (SBP, mmHg), diastolic blood pressure (DBP, mmHg), mean arterial pressure (MAP, mmHg), heart rate (HR, beats/min), maximal rate of rise of left ventricular pressure (+ dp/dt_max_) and maximal rate of fall of left ventricular pressure (−dp/dt_max_) at the baseline before ischemia, ischemia for 30 min and reperfusion for 1 h and 2 h, were measured. Triplicate measurements were taken and average values were used as the final result.

### Detection of cardiac function

Two weeks after I/R treatment, sixty rats were anaesthetized with isoflurane in supine position. A Vevo 770 high resolution imaging system ultrasonic apparatus (Visualsonics, Toronto, Canada) with RMV 704 probe frequency of 40 MHz was used to measure cardiac function. The left ventricular papillary muscle horizontal two-dimensional left ventricular short axis section was used to examine left ventricular endsystolic diameter (LVESD), left ventricular end diastolic diameter (LVEDd), left ventricular ejection fraction (LVEF) and left ventricular fraction shortening (LVFS). Four consecutive cardiac cycles were measured and the average value was used for statistical analysis.

#### Specimen preservation

The collected hearts were placed in precooled saline immediately after sacrificing the rats. The left ventricular anterior wall myocardial tissue 2 mm near the LAD ligation was cut off. A portion of the specimen was stored at −80°C and later used for qualitative real-time polymerase chain reaction (qRT-PCR) and western blot. A portion of the specimen was used to prepare tissue slices for fluorescence imaging. The remaining tissue was fixed in 10% formalin for 24 h and embedded in paraffin wax for TUNEL assay to test for apoptosis. The transfection efficiencies of miR-320 inhibitors lentivirus, miR-320 mimics lentivirus and ad-IGF-1 recombinant adenovirus were observed for further experiment.

The article "Down-regulation of microRNA-320 suppresses cardiomyocyte apoptosis and protects against myocardial ischemia and reperfusion injury by targeting IGF-1" was retracted in 2025. Reasons: plagiarized images; duplicated images; overlap with other authors' work; concerns about the authorship.

### Determination of MI size

At the end of the reperfusion hearts were quickly removed, washed with cold saline and placed at −20°C for 10 min and cut into 2 mm thick slices and placed into 1% triphenyl tetrazolium chloride at 37°C for 15 min. Slices were fixed in 4% formaldehyde for 24 h each heart slice was photographed with a digital camera and the left ventricle weight (LVW) was measured. LV, area at risk (AAR) and MI sizes were calculated using HPIAS-2000 image analysis software. The infarct size weight (ISW) was calculated using the following formula: ISW = (A1 * W1) + (A2 * W2) + (A3 * W3) + (A4 * W4) + (A5 * W5), where A is the percentage of MI size to LV size, W is the weight of the heart slices, and 1-5 indicate heart slice number. AAR weight (AARW) was calculated using the same method. The area of ischemic tissue is expressed with AARW/LVW×100, and the area of MI is expressed with ISW/AARW×100.

### Myocardial apoptosis detected by TUNEL

Tissue sections were deparaffinized and gradient washed with ethanol. Proteinase K solution was added and the samples were incubated at room temperature for 30 min. The sample was incubated for another 10 to 30 min at room temperature after adding 100 μl of equilibration buffer containing terminal deoxynucleotidyl transferase (TdT). Then, 5 μl of TdT solution and 45 μl of fluorescein labeled dUTP were added to each sample and mixed thoroughly. The TUNEL reaction solution was prepared according to the amount of samples. For the sham group, only fluorescein labeled dUTP was added, with no TdT. Finally, the samples were sealed and covered with reaction solution and incubated for 60 to 90 min at 37°C. Labeled apoptotic cells were analyzed under a green fluorescence excitation wavelength of 465 to 495 nm.

### Rat cardiomyocyte separation, culture and grouping

Healthy female Wistar rats were used to separate rat cardiomyocyte as follows: Amobarbital sodium (40 mg/kg) and heparin (250 μg/kg) were intraperitoneally injected into the rats. The rat chests were then opened and hearts were cut out 3-4 mm away from the heart root with the aortas reserved. The hearts were immediately put into a 750 μM Ca^2+^ solution at 37°C to discharge all the blood in the heart chambers. The aortic root was fixed to the mouth of a Langendorff perfusion tube, the flow rate was set to 9 mL/min/g, and the heart was perfused with oxygenated 750 μM Ca^2^^+^ solution at 37°C for 2 min, 100 μM Ca^2+^ free ethylene glycol tetraacetic acid solution for 4 min, and 0.1% II collagen enzyme solution for 10-15 min. The perfused heart was cut from the aortic root and the myocardium was cut from the heart bottom to the tip. Circulatory II collagen enzyme solution containing 1% bovine serum albumin (BSA) was added into the myocardium and the mixture was digested at 37°C, and filtered into a sterile tube through a 200 mesh nylon screen. The filtration was repeated 4-5 times. The filtered cell solution was subjected to natural subsidence at 37°C in a water bath, the supernatant was discarded, and cells were washed 3 times with enzyme elution and 2 times with medium M199. Laminin was used to pretreat 6-well plates at 37°C for 30 min. Cells were spread on the plates with a density of 10^4^/cm^2^, serum-free M199 medium was added to culture the cells for 3 h, removed non-adherent cells, and M199 medium was added again and the cells were cultured overnight. The cells were divided into eight groups: 1) Control group: cells were cultivated in normoxic condition; 2) H/R group: cells were subjected to 10 hours of hypoxia and 2 h of reoxygenation; 3) H/R + negative control (NC) group: cells were transfected with NC (an empty vector) and subjected to 10 h of hypoxia and 2 h of reoxygenation; 4) H/R + miR-320 inhibitor group: cells were transfected with 50 nM miR-320 inhibitors and subjected to 10 h of hypoxia and 2 h of reoxygenation; 5) HR + ad-IGF-1 group: cells were transfected with ad-IGF-1 and subjected to 10 h of hypoxia and 2 h of reoxygenation; 6) H/R + miR-320 mimics+ ad-IGF-1 group: cells were transfected with ad-IGF-1 and subjected to 10 h of hypoxia and 2 h of reoxygenation; 7) Control + miR-320 inhibitors group: cells were cultured under normal oxygen condition after transfected with miR-320 inhibitors lentivirus; and 8) Control + miR-320 mimics + ad-IGF-1 group: cells were cultured under normal oxygen condition after transfected with miR-320 inhibitors and ad-IGF-1 lentivirus. Cells at 50%-60% confluence were transfected using Lipofectamin 2000 (Invitrogen) cells were collected for analysis. All experiments were repeated three times.

The article "Down-regulation of microRNA-320 suppresses cardiomyocyte apoptosis and protects against myocardial ischemia and reperfusion injury by targeting IGF-1" was retracted in 2025. Reasons: plagiarized images; duplicated images; overlap with other authors' work; concerns about the authorship.

### H/R treatment

The H/R treatment in myocardial cells was based on the H/R model published by Ekhterae D *et al* [37]. Thirty minutes before H/R treatment, simulated ischemia and hypoxia medium containing no serum or glucose was prepared and was equilibrated using mixed low oxygen gas (95% N_2_ and 5% CO_2_) for more than 2 h. The normal myocardial cell medium was discarded and replaced with ischemia and hypoxia medium, and the myocardial cells were cultured in a hypoxia incubator (95% N_2_ and 5% CO_2_) at 37°C for 10 h to induce hypoxia. After cardiomyocytes were cultured in a hypoxia incubator for 10 h, the ischemia and hypoxia medium was discarded and DMEM medium containing glucose and 10% fatal bovine serum (FBS) was replaced. The cardiomyocytes were cultured in an incubator (95% air and 5% CO_2_) at 37°C for 2 h for reoxygenation.

### Annexin V/propidium iodide (PI) apoptosis assay

AnnexinV/PI assay was used to detect apoptosis. Rat myocardial cells were trypsinized and washed twice with phosphate buffered saline (PBS). Cells (1 to 5 × 10^5^/ml) were collected, washed twice with l mL PBS and centrifuged at 2000 rpm for 5 min. The cells were suspended in 500 μl of Binding Buffer and mixed with 5 μl AnnexinV-Fluorescein isothiocyanate (FITC) and 5 μl PI. The reaction was performed in the dark at room temperature for 5 to 15 min and analyzed within 1 h. Green fluorescence of AnnexinV-FITC was detected by FITC channel (FL1) and red fluorescence of PI by PI channel (FL3). Flow cytometry (488 nm excitation wavelength) detected FITC fluorescence with a bandpass filter (515 nm wavelength) and PI fluorescence was detected using a filter with a wavelength greater than 560 nm. Cell apoptosis was displayed by scatterplot with the lower left quadrant (FITC-/PI-) indicating healthy living cells, lower right quadrant (FITC+/PI-) indicating early apoptotic cells and upper right quadrant (FITC+/PI+) indicating necrosis and late apoptotic cells.

### qRT-PCR to detect miR-320 and IGF-1 mRNA

Trizol reagent was used to extract total RNA from tissue and cell samples, a UV spectrophotometer was used to measure the purity and concentration of RNA and the RNA integrity was verified by agarose gel electrophoresis. Taqman® RNA reverse transcription kit (Applied Biosystems) was used for reverse transcription of miR-320 and IGF-1 mRNA and the corresponding primer sequences are listed in Table 3. RT-PCR reaction (miR-320) included 1.0 μL cDNA, 1.0 μL forward primer (final concentration 100 nM), 1.0 μL reverse primer (final concentration 100 nM), 0.5 μL 10 × SYRB Green I, 10 μL 2 × PCR mix, diethyl pyrocarbonate (DEPC)-treated water to 20 μL. Reaction conditions (miR-320) were: initial denaturation at 95°C for 10 min, and 40 cycles of denaturation at 95°C for 15 s and annealing at 60°C for 1 min. PCR reaction (IGF-1 mRNA) was: 2.0 μL cDNA, 12.5 μL 2 × PCR mix, 1 μL forward primer (final concentration 100 nM), 1 μL reverse primer (final concentration 100 nM), DEPC-treated water added to 25 μL. Reaction conditions (IGF-1 mRNA) were: 32 cycles of denaturation at 94°C for 45 s, annealing at 52°C for 45 s, and extension at 72°C for 5 s. Specificity of the PCR reaction was confirmed by melting curve and 3.5% NuSieve agarose gel electrophoresis. Opticon Monitor software (version 3.0, BioRad) was used to analyze the PCR products. The threshold was manually set at the lowest point of the parallel rise of the amplification curve to obtain the Ct value of each reaction. Data were analyzed by 2^−ΔΔCt^ method.

The article "Down-regulation of microRNA-320 suppresses cardiomyocyte apoptosis and protects against myocardial ischemia and reperfusion injury by targeting IGF-1" was retracted in 2025. Reasons: plagiarized images; duplicated images; overlap with other authors' work; concerns about the authorship.

**Table 3:** Primer sequences of miR-320, IGF-1mRNA, U6 and GAPDH

Gene	Primers sequences
miR-320	F: 5′-ACACTCCAGCTGGGAAAAGCTGGGTTGAGA-′3
	R: 5′-ACACTCCAGCTGGGTCGCCCTC-′3
U6	F: 5′-CTCGCTTCGGCAGCACA-′3
	R: 5′-AACGCTTCACGAATTTGCGT-′3
IGF-1	F: 5′-AACTTTCTTTCCGTGCTG-′3
	R: 5′-TTCTGTCTATCGGTATGTTAC-′3
GAPDH	F: 5′-TATCGGACGCCTGGTTAC-′3
	R: 5′-CGTTCAAGTTGCCGTGTC-′3

Note: IGF-1, insulin like growth factor-1; miR-320, microRNA-320; GAPDH, glyceraldehyde phosphate dehydrogenase; F, forward; R, reverse.

### Western blotting

Approximately 0.25 g of tissue was placed into protein lysis buffer (Pik-day Biotechnology Research Institute, Beijing, China) and the sample was sonicated up and down six times, with each time for 1 min at 4°C and centrifuged. The supernatant was collected and stored at −70°C. Bradford assay was used to estimate protein concentration. SDS-PAGE gel electrophoresis (Pik-day Biotechnology Research Institute, Beijing, China) was used for protein separation and the separated proteins were transferred onto nitrocellulose membranes and blocked with 5% skim milk for 3 h. The membranes were incubated at 37°C for 1 h with diluted primary antibodies purchased from Cell Signaling Technology (Insulin-like growth factor 1 (IGF-1) (1 : 5000), IGF-1R (1 : 1000), p-IGF-1R (1 : 1000), total-apoptosis signal-regulating kinase 1 (total-ASK1) (1 : 2000), total-c-Jun N-terminal kinase (total-JNK) (1 : 1000), total-p38 (1 : 2000), phosphorylated-ASK1 (p-ASK1) (1 : 1000), p-JNK (1 : 1000), p-p38 (1 : 2000), B-cell lymphoma 2 (Bcl-2) (1 : 1000), Bax (1 : 2000), Caspase-3 (1 : 5000), β-actin (1 : 1000)). Goat anti-rabbit antibody (Sigma) was used as the secondary antibody (1 : 2000) and the membranes were incubated at 37°C for 45 min. ECL chemiluminescence reagent (Amersham Pharmacia Biotech) was exposed for 1 min, 5 min and 45 min, respectively, and then used to develop the reaction and wash. β-actin was used as an internal control. The western blot results were scanned and IPP 6.0 image analysis software was used to analyze the gray value of each band area to quantify the results. PBS was replaced as a negative control, and the purified target protein was used as a positive control.

The article "Down-regulation of microRNA-320 suppresses cardiomyocyte apoptosis and protects against myocardial ischemia and reperfusion injury by targeting IGF-1" was retracted in 2025. Reasons: plagiarized images; duplicated images; overlap with other authors' work; concerns about the authorship.

### Statistical analysis

SPSS19.0 statistical software was used for data analysis and measurement data were presented as mean ± standard deviation and tested by normality test. The *t-*test was used to compare differences between two groups and One-Way ANOVA analysis was employed to compare differences among groups (homogeneity of variance test was conducted before analysis). Pairwise LSD-*t* test was used to compare mean value of multiple groups. A two-sided *P* < 0.05 was considered statistically significant.
